# Rare Case of *Aspergillus ochraceus* Osteomyelitis of Calcaneus Bone in a Patient with Diabetic Foot Ulcers

**DOI:** 10.1155/2015/509827

**Published:** 2015-05-12

**Authors:** Farhang Babamahmoodi, Tahereh Shokohi, Fatemeh Ahangarkani, Mojtaba Nabili, Elham Afzalian Ashkezari, Sosan Alinezhad

**Affiliations:** ^1^Antimicrobial Resistance Research Center, Department of Infectious Diseases, Mazandaran University of Medical Sciences, Sari 47656-86143, Iran; ^2^Invasive Fungi Research Center, Department of Medical Mycology and Parasitology, Mazandaran University of Medical Sciences, Sari 48471-91971, Iran; ^3^Student Research Committee, Mazandaran University of Medical Sciences, Sari, Iran; ^4^Iranian Social Security Organization, Khatamolanbia Hospital, Gonbad-e Kavus 4971947953, Iran

## Abstract

Diabetes is the most common metabolic disease in humans. One of the major complications of the disease is foot ulcer that is prone to infection. The most common causes of infection which have been reported in these patients are bacteria and fungi such as *Candida, Aspergillus, and Rhizopus* species. We report one such rare case with calcaneal osteomyelitis caused by *Aspergillus ochraceus* in a patient with diabetic foot osteomyelitis. The case was a 68-year-old male with a history of type II diabetes for 2 years. The patient had two ulcers on the right heel bones for the past 6 months with no significant improvement. One of the most important predisposing factors to infectious diseases, especially opportunistic fungal infection, is diabetes mellitus. *Aspergillus* species can involve bony tissue through vascular system, direct infection, and trauma. Proper and early diagnosis and treatment of diabetic foot infection can reduce or prevent complications, such as osteomyelitis and amputation. The annual examination of feet for skin and nail lesion, sensation, anatomical changes, and vascular circulation can be useful for prevention and control of infection.

## 1. Introduction

Foot infections are the most common infection problem in diabetic patients that needs hospitalization and surgical intervention and it occurs in 10% of all patients with diabetes. Many studies show that diabetes mellitus is an important underlying disease for opportunistic fungal infections especially in diabetic foot osteomyelitis (DFO) patients [1]. These patients are vulnerable to fungal infections, which can be chronic and generalized and barely respond to antifungal therapy. Among fungal infections, candidiasis and aspergillosis are the most common factors and usually do not respond to antibiotic therapy and the disease becomes chronic [2]. There are many types of complications in DFO patients. That is present in approximately 20% of cases of foot infection in persons with diabetes [3] and greatly increases the likelihood that the patient will require a lower-extremity amputation [4]. One of the most controversial issues confronting the DFO is lack of widely agreed guidelines for its diagnosis, treatment, and management [5]. Almost all DFO cases result from contiguous spread of infection from adjacent soft tissue. The soft-tissue infection usually starts as a complication of a neuropathic ulcer but can result from penetrating injury or ischemic soft-tissue loss. Arterial insufficiency may be present but tends to play a less important role than neuropathy. As foot ulcer in diabetic patients is formed at the site of pressure such as great toes, metatarsal heads, and calcaneus, thus osteomyelitis most commonly affects the underlying bone of these sites. The midfoot bones are less commonly involved unless foot deformity has caused ulceration [6]. DFO can be caused by* Aspergillus* in immunosuppression and diabetes patients, but* Aspergillus* osteomyelitis is infrequently reported [7]. We reported one such rare case with calcaneal osteomyelitis caused by* A. ochraceus* in a patient with diabetic foot ulceration (DFU).

## 2. Case Presentation

In November 2014, a 68-year-old male, with a history of type II diabetes for 2 years and two ulcers on the right heel bones for the past 6 months, was admitted to an infection ward of Razi Hospital, Mazandaran, Iran. During the 6 months, the patient was hospitalized two times, but there was no significant improvement. On physical exams, there were two wounds on the right heel bones with erythema, soft-tissue swelling, tenderness, and discharge from the wounds. The wounds measured 2 × 3 cm and 2 × 2 cm (Figure 1). The patient noted occasional fever 1 week before admission. There were no other symptoms such as chest pain, cough, and sputum. In routine blood tests, no leukocytosis was detected, Hb was 8.4 g/dL, and ESR was 94 mm/hr. An ultrasound examination of the right foot has revealed soft-tissue swelling with irregular margins. Then magnetic resonance imaging (MRI) of right foot was performed. The MRI showed a destructive lesion in posterior part of calcaneus with soft-tissue involvement secondary to calcaneal osteomyelitis with abscess bone and soft tissue. Soft-tissue edema around ankle and hind foot due to inflammation is shown (Figure 2).

Finally, an excisional biopsy was performed for diagnosis of chronic osteomyelitis. The samples were sent to the laboratory for detection of atypical mycobacteria, fungi, and pathological condition. The pathology finding in H&E staining was chronic inflammatory cells and fungal septate hyphae. Bacterial cultures were negative. In direct microscopic examination (KOH + DMSO preparation) of the biopsy specimen dichotomous branching septate hyphae and rough globose conidia were observed (Figure 3). The biopsy from bone specimens was cultivated in Sabouraud dextrose agar (SDA) and brain heart infusion agar (BHIA). SDA and BHIA culture media after 72 hours' incubation at 27°C yielded yellow-orange colonies with granular texture, and the reverse was pale to brownish. Microscopic morphology of colony shows conidial heads that were radiating and splitting into several columns. Conidiogenous cells were biseriate. Conidiophores were brownish and roughened near the vesicle. Conidia were globose to subglobose, pale green, and finely echinulate. Presumptive identification primarily on the basis of its macroscopic and microscopic characteristics was as* Aspergillus flavus* (Figure 4).

The polymerase chain reaction assays have been performed with the yielded colonies. A part of *β*-tubulin gene was amplified using primer pair Bt-F (5′-GGTAACCAAATCGGTGCTGCTTTC) and Bt-R (5′-ACCCTCAGTGTAGTGACCCTTGGC) and sequenced for accurate identification [8]. The comparative DNA sequences analysis by nucleotide Basic Local Alignment Search Tool (BLAST) showed that the amplified sequence had 99% identity with the beta-tubulin genes of* A. ochraceus* with GenBank accession number FR775371.1.

According to the criteria of EORTC/MSG (European Organization for Research and Treatment of Cancer/Mycoses Study Group), the present case was a proven invasive aspergillosis [9].* Aspergillus* osteomyelitis was diagnosed based on positive direct microscopy, culture, and histological data. In KOH preparation and histopathology examinations of wound biopsy hyphae are accompanied by evidence of associated tissue damage, as well as recovery of* Aspergillus* colonies in culture of a specimen obtained using a sterile procedure and MRI finding of abnormal site consistent with an invasive process. Antifungal susceptibility testing of the isolate was performed by microbroth dilution technique in accordance with Clinical and Laboratory Standard Institute (CLSI) guidelines M38-A2 [10]. Antifungal susceptibility of isolated* Aspergillus* showed low minimum inhibitory concentrations of posaconazole (Schering-Plough, Kenilworth, USA) (0.032 *μ*g/mL) and caspofungin (Merck Sharp & Dohme, Haarlem, Netherlands) (0.125 *μ*g/mL). Voriconazole (Pfizer Central Research, Sandwich, United Kingdom) (1 *μ*g/mL), itraconazole (Janssen Research Foundation, Beerse, Belgium) (1 *μ*g/mL), and amphotericin B (Bristol-Myers Squibb, Woerden, Netherlands) (16 *μ*g/mL) showed reduced susceptibility. He was primarily before accessing the antifungal susceptibility test treated with amphotericin B (deoxycholate) 50 mg/d. Finally, the treatment regimen was shifted to oral voriconazole 200 mg 2 times per day and patient was discharged with good general condition. The patient's signs (two wounds on the right heel bones) improved after treatment for 4 months by voriconazole (Figure 5).

## 3. Discussion

Patients with diabetes mellitus are at risk for infectious diseases, especially opportunistic fungal diseases. People with diabetes are prone to having fungal diseases for various reasons such as progressive suppression of immune system and increasing glucose concentration in mucosal tissues and various body fluids. So many reports show increasing of prevalence and severity of fungal infections in mouth, genital systems, nail, urinary system, and tissues, especially in patients with incompletely treatment. Foot in diabetic patients is a high risk organ for trauma and neuropathy that is prone to fungal infections [11, 12]. Fungi such as* Aspergillus* conidia are known to be ubiquitous in nature and are the commensals in the respiratory tract. In patients with immunosuppression, these organisms can multiply and cause widespread infection involving respiratory system and sometimes even skeletal system. Fungal osteomyelitis is increasingly reported in the literature but* Aspergillus* osteomyelitis is infrequently reported. Osteomyelitis is common in cases of polytrauma, where multiple surgeries cause a break in the natural barriers of skin and mucous membrane, and compromises the patient's immune system. In such cases* Staphylococcus aureus* is the most common cause and the long bone metaphysis is the most common localization of osteomyelitis. However, fungi, anaerobes, and so forth are rare causative agents and involvement of calcaneus bone is infrequent condition [13, 14]. Koehler et al. reviewed 47 bones and joints cases infected by aspergillosis and* A. fumigatus* was the most common* Aspergillus* species. The osteomyelitis of the foot bones was reported as 5% and a total of 38% of cases had disseminated aspergillosis with initial presentation of local symptoms but in our patient there were only local symptoms (lung and brain CT scans were normal) [15]. Similar to Bathoorn et al. and Koehler et al. study, in our study voriconazole was used in treatment [16].

*Aspergillus ochraceus* is a mold species in the genus* Aspergillus* known to produce the toxin ochratoxin A, one of the most abundant food-contaminating mycotoxins, and citrinin. It also produces the dihydroisocoumarin mullein [17].

*Aspergillus* can involve bony tissue through vascular system, direct infection, and trauma. Generally, one of the common fungal diseases which occurred in uncontrolled diabetes mellitus is mucormycosis. Mucormycosis is the common name given to several different diseases caused by fungi of the order Mucorales. Usually mucormycosis presents as an acute infection and manifests in rhinocerebral, pulmonary, gastrointestinal, cutaneous, or disseminated forms, rarely affecting otherwise healthy people [18].

Proper and early diagnosis and treatment of diabetic foot infection can reduce period and complication, such as osteomyelitis and amputation. Two parameters should be determined for this purpose: (1) the causative organisms and (2) wound size. Microbiological examinations of biopsy material are necessary for identification of the infectious organisms to species level and determining in vitro susceptibility profile to antifungal that can assist clinicians in treatment decision making. Some methods such as radiography, isotope scan, CT scan, and MRI can be useful for measurement of wound extent which have advantages and disadvantages of their own [19]. Amputation in patients with DFU can occur due to missing diagnosis of osteomyelitis. Hematologic variables such as WBC count and ESR level may not be helpful in making the diagnosis. Though normal range of ESR reduces probability of osteomyelitis and with ESR of more than 70 mm/hr, the diagnosis of osteomyelitis is more likely. But biopsy of the bone is necessary for definitive diagnosis of DFO [20]. In our patient, ESR level was 94 mm/hr which increased the likelihood of osteomyelitis.

Other points that should be considered regarding osteomyelitis are as follows: lack of healing after a few weeks while the wound is well protected and the pressure is removed, radiographic evidence of bone lesion, unexplained leukocytosis, and wound with surface more than 2 cm and depth of more than 3 mm can be suspected to osteomyelitis [21]. Both of the wounds surfaces were greater than 2 cm^2^. MRI shows extent of the wound more than other methods. CT scan and ultrasound are helpful for diagnosis of soft-tissue lesions such as abscess, fistula, and involvement cortex of the bone [22].

*Aspergillus* can easily infect damaged foot tissue in diabetic patients through contaminated shoes and clothes. So using proper shoes and clothes and also the periodical examination of the feet for detecting skin and nail lesion, sensation of foot, anatomical changes, and vascular circulation of foot can be useful for prevention of infection [23].

Cases of fungal osteomyelitis in the literature that were reviewed showed that surgical resection accompanied by systemic antifungals therapy had a lower recurrence and higher success rate as compared to those that were treated with antifungals alone, which may be due to the fact that penetration of most drugs into the bone tissue is low [24]. We treated our patient with surgical debridement along with amphotericin B and voriconazole with good results.

This report highlights the presence of emerging pathogens and supports the necessity of careful microbiological identification at the species level, thereby reinforcing the physician's attention toward the possibility of invasive fungal infection in diabetic patients.

## Figures and Tables

**Figure 1:** Two wounds on the right heel bones.

**Figure 2:** The MRI showed a destructive lesion in posterior part of calcaneus.

**Figure 3:** A direct examination of the removed fungus ball showing septate and dichotomous branching hyphae, vesicles, and conidia suggestive of* Aspergillus* species (KOH + DMSO preparation, ×800).

**Figure 4:** Conidial heads and brownish roughened conidiophores of* Aspergillus ochraceus* (Lactophenol Aniline Blue preparation).

**Figure 5:** The complete remission of right heel lesion after 4-month treatment with voriconazole.

## References

[1] Aly F. Z., Blackwell C. C., MacKenzie D. A. C. (1991). Chronic atrophic oral candidiasis among patients with diabetes mellitus—role of secretor status. *Epidemiology & Infection*.

[2] Mlinariæ-Missoni E., Kaleniæ S., Vukeliæ M., de Syo D., Belicza M., Vaziæ-Babiæ V. (2005). Candida infections in diabetic foot ulcers. *Diabetologia Croatica*.

[3] Grayson M. L., Gibbons G. W., Habershaw G. M. (1994). Use of ampicillin/sulbactam versus imipenem/cilastatin in the treatment of limb-threatening foot infections in diabetic patients. *Clinical Infectious Diseases*.

[4] Lavery L. A., Armstrong D. G., Wunderlich R. P., Mohler M. J., Wendel C. S., Lipsky B. A. (2006). Risk factors for foot infections in individuals with diabetes. *Diabetes Care*.

[5] Lipsky B. A. (2004). A report from the international consensus on diagnosing and treating the infected diabetic foot. *Diabetes/Metabolism Research and Reviews*.

[6] Lavery L. A., Harkless L. B., Ashry H. R., Felder-Johnson K. (1994). Infected puncture wounds in adults with diabetes: risk factors for osteomyelitis. *The Journal of Foot and Ankle Surgery*.

[7] Tew C. W., Han F. C., Jureen R., Tey B. H. (2009). Aspergillus vertebral osteomyelitis and epidural abscess. *Singapore Medical Journal*.

[8] Balajee S. A., Borman A. M., Brandt M. E. (2009). Sequence-based identification of *Aspergillus*, *Fusarium*, and *Mucorales* species in the clinical mycology laboratory: where are we and where should we go from here?. *Journal of Clinical Microbiology*.

[9] De Pauw B., Walsh T. J., Donnelly J. P. (2008). Revised definitions of invasive fungal disease from the European organization for research and treatment of cancer/invasive fungal infections cooperative group and the national institute of allergy and infectious diseases mycoses study group (EORTC/MSG) consensus group. *Clinical Infectious Diseases*.

[10] CLSI (2008). *Reference Method for Broth Dilution Antifungal Susceptibility Testing of Filamentous Fungi; Approved Standard*.

[11] Vazquez J. A., Sobel J. D. (1995). Fungal infections in diabetes. *Infectious Disease Clinics of North America*.

[12] Danowski T. S., Sabeh G., Sarver M. E., Shelkrot J., Fisher E. R. (1966). Shin spots and diabetes mellitus. *The American Journal of the Medical Sciences*.

[13] Roy M., Sidhom S., Kerr K. G., Conroy J. L. (2009). Case report: *Rhodococcus erythropolis* osteomyelitis in the toe. *Clinical Orthopaedics and Related Research*.

[14] Pattanashetty O., Dayanand B., Bhavi S. B., Bami M. (2013). Rare case of isolated *Aspergillus osteomyelitis* of toe: presentation and management. *Journal of Orthopaedic Case Reports*.

[15] Koehler P., Tacke D., Cornely O. A. (2014). Aspergillosis of bones and joints—a review from 2002 until today. *Mycoses*.

[16] Bathoorn E., Escobar Salazar N., Sepehrkhouy S., Meijer M., de Cock H., Haas P.-J. (2013). Involvement of the opportunistic pathogen *Aspergillus tubingensis* in osteomyelitis of the maxillary bone: a case report. *BMC Infectious Diseases*.

[17] Ghibaudo G., Peano A. (2010). Chronic monolateral otomycosis in a dog caused by *Aspergillus ochraceus*. *Veterinary Dermatology*.

[18] Sugar A. M., Mandell G., Douglas. R., Bennett J. (1990). Agents of mucormycosis and related species. *Principles and Practice of Infectious Diseases*.

[19] Höpfner S., Krolak C., Kessler S. (2004). Preoperative imaging of charcot neuroarthropathy in diabetic patients: comparison of ring PET, hybrid PET, and magnetic resonance imaging. *Foot and Ankle International*.

[20] Hartemann-Heurtier A., Senneville E. (2008). Diabetic foot osteomyelitis. *Diabetes & Metabolism*.

[21] Lavery L. A., Armstrong D. G., Peters E. J. G., Lipsky B. A. (2007). Probe-to-bone test for diagnosing diabetic foot osteomyelitis: reliable or relic?. *Diabetes Care*.

[22] Termaat M. F., Raijmakers P. G. H. M., Scholten H. J., Barker F. C., Patka P., Haarman H. J. T. M. (2005). The accuracy of diagnostic imaging for the assessment of chronic osteomyelitis: a systematic review and meta-analysis. *The Journal of Bone and Joint Surgery—American Volume*.

[23] Azizi F., Gouya M. M., Vazirian P., Dolatshahi P., Habibian S. (2003). The diabetes prevention and control programme of the Islamic Republic of Iran. *Eastern Mediterranean Health Journal*.

[24] De Vuyst D., Surmont I., Verhaegen J., Vanhaecke J. (1992). Tibial osteomyelitis due to *Aspergillus flavus* in a heart transplant patient. *Infection*.

